# High LINC01605 expression predicts poor prognosis and promotes tumor progression via up-regulation of MMP9 in bladder cancer

**DOI:** 10.1042/BSR20180562

**Published:** 2018-09-05

**Authors:** Zhiqiang Qin, Yi Wang, Jingyuan Tang, Lei Zhang, Ran Li, Jianxin Xue, Peng Han, Wei Wang, Chao Qin, Qianwei Xing, Jie Yang, Wei Zhang

**Affiliations:** 1 Department of Urology, The First Affiliated Hospital of Nanjing Medical University, Nanjing 210009, China; 2 Department of Urology, Jiangsu Province Hospital of TCM, Affiliated Hospital of Nanjing University of TCM, Nanjing 210029, China; 3 Department of Urology, Affiliated Hospital of Nantong University, Nantong 226001, China

**Keywords:** Bladder cancer, EMT, lncRNA LINC01605, MMP9, Migration

## Abstract

The advent of high-throughput sequencing methods has facilitated identification of novel long non-coding RNAs (lncRNAs), which have been demonstrated to play an important role in multiple tumors. Moreover, with the assistance of bioinformatics analysis, LINC01605 has been found to be up-regulated in bladder cancer (BC) tissues compared with normal tissues. Hence, the present study was to explore its specific biological role and related mechanism in BC. The relative expression level of LINC01605 was measured in a cohort of BC tissues with matched normal tissues as well as human BC cell lines by quantitative real-time PCR (qRT-PCR). Survival analysis was performed to explore the relationship between LINC01605 expression and the prognosis of BC patients. The biological function of LINC01605 was studied *in vitro*and *in vivo*, by means of CCK-8 assay, colony formation assay, transwell assay, and tumor xenografts mice model. LINC01605 was found to be frequently highly expressed in both human BC cells and tissues. Survival analysis indicated that high LINC01605 expression was associated with higher histological grade and clinical stages. In addition, down-regulated LINC01605 in BC cells could significantly inhibit the abilities of proliferation, migration, and invasion *in vitro* and knockdown of LINC01605 in subcutaneous xenograft tumor model could impede tumorigenesis *in vivo*. Mechanistically, LINC01605 could activate epithelial–mesenchymal transition (EMT) signaling pathway and promote the expression of matrix metallopeptidase (MMP) 9 (MMP9). In summary, our results shed light on that LINC01605, as a new prognostic biomarker, could promote the proliferation, migration, and invasion of BC cells via activating EMT signaling pathway and up-regulating MMP9 expression.

## Introduction

Bladder cancer (BC), characterized by frequent recurrence and high mortality, is one of the most common urologic malignancy over the world, with 79030 newly estimated cases and 16870 newly estimated deaths in U.S.A. in 2017 [1,2]. Although the majority of BCs are non-invasive (70–75%), they will metastasize over time and eventually progress to muscle-invasive disease (25–30%) [3]. Many known factors could lead to BC, such as elderly age, cigarette smoking, chemicals, occupational exposures, contact with carcinogens, and so on [4]. Despite a diversity of treatments used for BC, including surgery, chemo- or radiotherapy, the survival benefit remains to be limited and its incidence and mortality have gradually increased in the past decade [5]. Moreover, due to the absence of early warning signs, symptoms, and effective treatments, many patients would develop progression or metastases at the time of diagnosis and the 5-year survival rate of BC remains unsatisfied [6]. However, accurate mechanisms in the development and progression of BC remain unclear [7]. Therefore, there is an urgent need to improve understanding of tumor biology in BC and identify more effective and highly selective potential targetted therapeutic agents for BC treatment.

Long non-coding RNAs (lncRNAs), defined as non-coding RNAs longer than 200 nts in length, have captured significant attention in both normal biology processes and diseases including cancer [8–12]. Accumulating evidence have demonstrated that the function of lncRNAs could be either as an oncogene, or a tumor suppressor gene, or both involved in tumor prognosis and progression, depending on the circumstance(s) [13–15]. Amongst them, many lncRNAs, such as MALAT1, H19, and HOTAIR have been demonstrated as a critical regulator of carcinogenesis and development of many cancers [16–18]. The advent of high-throughput sequencing methods as well as microarray analysis has facilitated identification of novel lncRNAs, which have been demonstrated to play an important role in multiple tumors [19]. Linc01605, a 4981-kb lncRNA (also named as LincDUSP), located at chromosome 8p11.23, was found to be highly expressed in BC tissues compared with normal tissues through bioinformatics analysis. However, the molecular mechanisms that dictate and govern the role of LINC01605 in tumor progression have not been well elucidated so far.

Matrix metallopeptidases (MMPs) as an important group of zinc-dependent proteolytic enzymes, are capable of degrading components of the extracellular matrix and other barriers, amongst which, MMP2 and MMP9 are found to mainly cleave collagen IV in the basement membrane to promote cell invasion in cancer cells [20,21]. Accumulating researches had demonstrated that MMP9 was highly expressed in many human tumors and it was significantly associated with poor survival in cancer patients by means of promoting the invasion of cancer cells [22–24].

The focus of this research was to identify the possible relationship between LINC01605 and BC and to uncover its potential mechanisms. Meanwhile, this was the first time for us to evaluate the expression of LINC01605 in BC and explore its clinical significance by *in vitro* and *in vivo* models. Thus, LINC01605 could be a new molecular biomarker or a novel target for the treatment of BC in the future study.

## Methods

### The Cancer Genome Atlas data acquisition

We downloaded genomic alteration data on patients with BC and corresponding clinicopathologic profiles at The Cancer Genome Atlas (TCGA; https://cancergenome.nih.gov/), which as a freely opened public platform, is a source for abundant cancer-related data [25]. This study complied with TCGA publication guidelines and policies (http://cancergenome.nih.gov/publications/publicationguidelines). Thus, the relevant expression level and survival curves of LINC01605 in BC of TCGA database were determined.

### Patients and BC samples

Ninety-two pairs of frozen BC tissues and matched normal tissues were obtained from the Department of Urology of The First Affiliated Hospital of Nanjing Medical University from February 2009 to August 2014 with appropriate informed consent. The follow-up deadline was August 2017. All the tissues were stored at −80°C before RNA isolation and matched normal bladder tissues were above 3 cm away from cancer. The diagnosis was verified by histopathological examination and the assessment was conducted by quantitative real-time PCR (qRT-PCR) and Western blot. All of the patients’ data (*n*=92) had been collected as clinicopathologic characteristics of BC and survival rate. The present study was approved by the Institutional Research Ethics Committees of the First Affiliated Hospital of Nanjing Medical University.

### qRT-PCR

Total RNA from the clinical samples and cultured cell lines were extracted with TRIzol reagent (Invitrogen, U.S.A.) and their relative cDNA was synthesized by Primescript RT Reagent (TaKaRa, Japan) according to the manufacturer’s instructions. All qRT-PCR were performed by using StepOne Plus Real-Time PCR system (Applied Biosystems, U.S.A.) with SYBR^®^ Premix ExTaq™ Reagent (TaKaRa, Japan). The following primers were used for qRT-PCR:

LINC01605, Forward: 5′-CGTTACAAACAGCCGACCTT-3′
Reverse: 5′- CCAGGGAGGGACTCAAGAAT-3′
β-actin, Forward: 5′-CCTGGCACCCAGCACAAT-3′
Reverse: 5′-GCTGATCCACATCTGCTGGAA-3′

Data analysis was performed with ABI Step One Software version 2.1 and the relative mRNA level was calculated using 2^−ΔΔ*C*^_t_ methods.

### Cell culture

The human BC cell lines (EJ, T24, 253j, J82) and human normal uroepithelial cells (SV-HUC-1) were obtained from the American Type Culture Collection (ATCC, U.S.A.). The cells were cultured in DMEM medium supplemented with 10% FBS (Gibco, U.S.A.) and 1% penicillin/streptomycin (Invitrogen, U.S.A.). They were maintained in a humidified incubator at 37°C in 5% CO_2_ atmosphere.

### Western blot

Cells or frozen tissues were lysed in cell lysis buffer for 30 min on ice and centrifuged at 14000 ***g*** at 4°C for 15 min. The total protein concentration was calculated by the BCA Protein Assay kit (Pierce, U.S.A.). Proteins were separated by SDS/PAGE (10% gel) and transferred on to a PVDF membrane (Millipore, U.S.A.). Western blot analysis followed a standard procedure. The primary antibodies (N-cadherin, Vimentin, β-catenin, MMP9, and GAPDH) were obtained from Cell Signaling Technology, U.S.A. The anti-mouse and anti-rabbit secondary antibodies were also from Cell Signaling Technology, U.S.A.

### Transfection

Lentivirus packaging cells were transfected with LV3-pGLV-h1-GFP-puro vector (GenePharma, China) containing either the LINC01605 knockdown (sh-lnc01605-1 and sh-lnc01605-2) or LINC01605 overexpression (Lnc01605) and a negative control sequence (NC), respectively. Lentiviral transduction was performed in EJ and T24 cell lines. Pools of stable transductants were generated by selection using puromycin (4 μg/ml) for 2 weeks.

### Cell proliferation assay

The CCK-8 assay (Dojindo Laboratories, Japan) was used to estimate the proliferation potential. Cells were seeded in 96-well plates with 3000 cells/well. CCK-8 reagents were added into wells after cells were grown for 1, 2, 3, and 4 days, respectively and the absorbance was measured at 450 nm using a microplate reader at 2 h after CCK-8 addition.

### Colony formation assay

Cells transfected with the indicated vectors were seeded into six-well plates (600 cells/well) and cultured in medium containing 10% FBS for 2 weeks. Then, the colonies were fixed with paraform for 1 h and stained with 0.1% Crystal Violet for anther 1 h. The colonies were counted under the microscope and each group was repeated three times.

### Transwell cell migration and invasion assay

The assay of cell migration or invasion was conducted by a 24-well Transwell chamber (Costar, U.S.A.) with or without Matrigel (Invitrogen, U.S.A.). Cells (2 × 10^4^) were seeded into the upper chambers with serum-free medium and the chambers would be inserted into the 24-well plate. Medium containing 10% FBS was added to the lower chamber. Cells were incubated at 37°C with 5% CO_2_ atmosphere for 48 h and then cells on the surface of the upper chambers that did not migrate through the pores were removed with a cotton swab. Meanwhile, cells which migrated to the bottom surface of the chamber were fixed with paraform for 1 h and stained with 0.1% Crystal Violet for another 1 h. Number of migratory and invasive cells were counted in five randomly selected fields under the microscope and the presented data represented three individual experiments.

### Xenograft studies

The animal experiments were carried out based on the Guide for the Care and Use of Laboratory Animals published by the U.S. National Institutes of Health (NIH publication number 85e23, revised 1996) and it was performed at Animal Experiment Center of The First Affiliated Hospital of Nanjing Medical University. Related animal ethics authorization was approved by the Animal Research Ethics Committee of Nanjing Medical University. The 5-week-old female nude mice were randomly divided into two groups consisting of five mice each. The stable cells (7 × 10^6^) sh-lnc01605-2-EJ and the control cells (NC-EJ) were suspended in 150-μl PBS and injected subcutaneously into the flank of each mouse. Tumor size was calculated (length × width^2^ × 0.52) once a week. After 6 weeks, tumors were removed, weighed, fixed, and embedded for immunohistochemical staining.

### Immunohistochemistry

The relative expression of Ki-67 protein was evaluated by immunohistochemistry performed on tissue microarray. With a primary antibody against Ki-67, tissue microarray was incubated at 4° C overnight and incubated with HRP–conjugated secondary antibody followed by DAB staining. The positive level of IHC staining was scored by two urologists and patients with different scores were divided into low- and high-staining groups. For assessing the association of lnc01605 expression with clinicopathologic characteristics of the BC patients, following parameters were included: gender (male and female), age (≤60 and >60 years), multiplicity (single and multiple), histological stage (low and high), lymph nodes metastasis (no and yes) and tumor stage (TNM stages Ta,T1, and T2-T4).

### Statistical analysis

Statistical analyses were conducted by SPSS 22.0 software. All the data were presented in the format of mean ± S.D. from three independent experiments at least. Student’s *t*test and the χ^2^ test were used to analyze differences between groups and survival curves were drawn by the Kaplan–Meier method. Moreover, *P*<0.05 was considered statistically significant.

## Results

### LINC01605 is highly expressed in BC of TCGA database and predicts poor prognosis

The expression level of LINC01605 was significantly up-regulated in BC clinical tissues compared with marched adjacent non-cancerous tissues (*P*=6.372e-08, Figure 1A). With regard to overall survival, patients with high LINC01605 expression had a significantly poorer prognosis than those with low LINC01605 expression (*P*=0.045, Figure 1B). These results above implied a potential role of LINC01605 as a novel biomarker for BC progression.

**Figure 1:** The expression level and survival curves of LINC01605 in BC of TCGA database (**A**) The level of LINC01605 expression in BC clinical tissues and marched adjacent non-cancerous tissues (*P*=6.372e-08). (**B**) Patients with high LINC01605 expression had a significantly poorer prognosis than those with low LINC01605 expression (*P*=0.045).

### LINC01605 is highly expressed in BC tissues and cell lines

To assess the expression level of LINC01605 with qRT-PCR in BC tissues, 20 pairs of BC tissues and adjacent pair-matched non-cancerous tissues were selected and the results suggested that LINC01605 expression was markedly up-regulated in mRNA level compared with the adjacent normal tissue (Figure 2A,B). To explore the mRNA expression of LINC01605 in BC cell lines, four human BC cell lines (EJ, T24, 253j, J82) and one normal human uroepithelial cells (SV-HUC-1) were selected for qRT-PCR. As displayed in Figure 2C, *LINC01605* mRNA was up-regulated by 13.4- to 19.3-fold in all BC cell lines compared with SV-HUC-1.

**Figure 2:** The expression level and survival curves of LINC01605 in BC cell lines and tissues (**A,B**) *LINC01605* mRNA expression in 20 pairs of BC tissues and marched adjacent non-cancerous tissues. (**C**) qRT-PCR of LINC01605 expression in BC cell lines and normal human uroepithelial cells (SV-HUC-1). (**D**) Kaplan–Meier survival curves of patients with BC based on LINC01605 expression conditions. The patients in the high expression group had a significantly more unfavorable prognosis than those in low expression group (*P*=0.0257, log rank test). Data represent the mean ± S.D. from three independent experiments, *P<0.05, **P<0.01

### LINC01605 expression is correlated with histological grade, clinical stage, and overall survival in BC patients

To validate the relationship between LINC01605 expression level and clinicopathologic features, 92 cases of BC tissues were enrolled for qRT-PCR. The mean expression level of LINC01605 in all BC tissues was used as a cut-off value and all samples were divided into a relatively low expression group (*n*=47) and a relatively high expression group (*n*=45). Although, no statistical correlation had been observed with gender (*P*=0.125), age (*P*=0.620), multiplicity (*P*=0.148), or lymph nodes metastasis (*P*=0.149), LINC01605 did present a significant correlation with histological grade (*P*=0.012) and TNM stage (*P*=0.032). In other words, a high level of LINC01605 expression was correlated with a higher histological grade or TNM stage, compared with the group of low expression (Table 1). As displayed in Figure 2D, we could find that high LINC01605 expression level in BC patients, had a significantly shorter overall survival than those with low expression (*P*=0.0257). All in all, all these data suggested the important role of LINC01605 in the development and progression of BC.

**Table 1:** Association of LINC01605 expression with clinicopathologic characteristics of BC patients

Parameters	Number of cases	lnc01605 expression		*P*-value
		Low	High	
Gender				0.125
Male	62	28	34	
Female	30	19	11	
Age (years)				0.620
<60	33	18	15	
≥60	59	29	30	
Multiplicity				0.148
Single	52	30	22	
Multiple	40	17	23	
Histological grade				**0.012**
Low	45	29	16	
High	47	18	29	
Lymph nodes metastasis				0.149
No	75	41	34	
Yes	17	6	11	
TNM stage				**0.032**
Ta,T1	39	25	14	
T2-T4	53	22	31	

### LINC01605 promotes cell proliferation *in vitro*

To further investigate the biological role of LINC01605 in BC cell lines, we stably knocked down or overexpressed LINC01605 expression by lentivirus-mediated shRNA transfection in two BC cell lines (EJ and T24). Meanwhile, the silenced cells were named as sh-lnc01605-1 or sh-lnc01605-2, respectively, the overexpressed cell lines were called Lnc01605 and the pair-matched control cells were named NC. As indicated in figures, the expression levels were respectively confirmed by qRT-PCR. These data demonstrated the effectiveness of the down- or up-regulated LINC01605 expression levels (Figure 3A,B,G,H, *P*<0.01).

**Figure 3:** Effect of LINC01605 on proliferation and growth of BC cell lines EJ and T24 (**A**,**B**) qRT-PCRs were used to verify the efficiency of LINC01605 knockdown. sh-lnc01605-1 and sh-lnc01605-2 indicate LINC01605 knockdown; NC indicate cells transfected with a empty vector. (**C**,**D**) Growth curve analysis showing the cell growth of EJ and T24 cells with LINC01605 knockdown. (**E**,**F**) The efficiencies of cell colony formation in EJ and T24 cells with LINC01605 knockdown. (**G**,**H**) qRT-PCR were used to verify the efficiency of LINC01605 overexpression (named as Lnc01605). (**I**,**J**) Growth curve analysis showing the cell growth of EJ and T24 cells with LINC01605 overexpression. (**K**,**L**) The efficiencies of cell colony formation in EJ and T24 cells with LINC01605 overexpression. Data represent the mean ± S.D. from three independent experiments, *P<0.05.

We could find from the growth curve analysis that down-regulation of LINC01605 could significantly inhibit cell growth (Figure 3C,D, *P*<0.05) and up-regulated LINC01605 expression could markedly enhance cell growth in EJ and T24 cells, compared with the control cells (Figure 3I,J, *P*<0.05). Meanwhile, a colony formation assay was performed simultaneously. Consistent with the results of CCK-8 assay, silenced or overexpressed LINC01605 expression could significantly inhibit or enhance colony-formation capacity of EJ and T24 cells (Figure 3E,F,K,L, *P*<0.05). All these data shed light on that LINC01605 may be involved in the regulation of cell proliferation in BC.

### LINC01605 promotes cell migratory and invasive potential

To examine the effect of LINC01605 silencing or overexpressing on regulating the ability of migration and invasion in BC cells, transwell migration and invasion assays were performed on EJ and T24 cells. As indicated in the results of transwell migration assays, knocking down LINC01605 could significantly reduce the migration capability of EJ and T24 cells, while overexpressing LINC01605 could significantly increase the ability of migration. Similar results could be found in the transwell invasion assays (Figure 4A–D, *P*<0.01**)**.

**Figure 4:** LINC01605 promotes cell migratory and invasive potential and its underlying mechanism (**A–D**) Transwell migration assay and Matrigel invasion assay in EJ and T24 cells with LINC01605 knockdown or overexpression. (**E**,**F**) N-cadherin, Vimentin, β-catenin, MMP9 protein expression levels were analyzed by Western blot in EJ and T24 cells with LINC01605 knockdown or overexpression. Data represent the mean ± S.D. from three independent experiments; **P<0.01.

To further explore the mechanism that LINC01605 affects the migration and invasion ability of BC cells, Western blot was conducted to examine the expression levels of N-cadherin, Vimentin, β-catenin, and MMP9, which were associated with regulating cell adhesion and metastasis. Western blot analysis demonstrated that LINC01605 down-regulation markedly suppressed the expression of N-cadherin, Vimentin, β-catenin, and MMP9 in EJ and T24 cell lines, while LINC01605 overexpression significantly increased their expression (Figure 4E,F). Meanwhile, the fold change was displayed below each lane. Taken together, all these data shed light on that LINC01605 could promote the migration and invasion ability of BC cells and the potential mechanism might be the down-regulation of adhesion and metastasis related molecules by activating epithelial–mesenchymal transition (EMT) signaling pathway.

### MMP9 interference reverses the malignant progress of LINC01605 on BC cells

To determine whether LINC01605 promotes BC progression through the regulation of MMP9 expression, we investigated the role of MMP9 by which it played in the cell function of BC cells. MMP9 small interference RNA (siMMP9) was transfected into EJ and T24 LINC01605 overexpression cells (Lnc01605) and the control cells (NC) to decrease endogenous MMP9 expression. According to the outcomes of CCK-8 assays, MMP9 knockdown resulted in a decreased cell growth of Lnc01605. Meanwhile, no statistical difference had been observed between the LINC01605+siMMP9 group and the NC group in EJ and T24 cell lines. Furthermore, when MMP9 knockdown totally, it could reverse the promoting effects of LINC01605 cell growth (Figure 5A). Similar results were also shown in transwell invasion assays, in the results of which, it exhibited that addition of siMMP9 into LINC01605 group could reduce the migration capability of EJ and T24 cells. Moreover, when MMP9 knockdown totally, it could significantly decrease the ability of migration (Figure 5B–E, *P*<0.01). On the other hand, Western blot analysis also presented that the levels of MMP9 were decreased in the group of siMMP9, compared with the group of Lnc01605 in EJ and T24 cell lines. Meanwhile, siMMP9 had a more decreased level than the group of Lnc01605+siMMP9 (Figure 5F). In summary, silencing MMP9 in LINC01605-overexpressed BC cells significantly increased its abilities of proliferation, migration, and invasion. In other words, we suggested that LINC01605 possibly promoted BC progression via the regulation of MMP9 expression.

**Figure 5:** MMP9 rescues the oncogenic role of LINC01605 in BC cells (**A**) Growth curve analysis showing the cell growth of EJ and T24 cells with LINC01605 overexpression and MMP9 knockdown. (**B–E**) Transwell migration assay and Matrigel invasion assay in EJ and T24 cells with LINC01605 overexpression and MMP9 knockdown. (**F**) MMP9 protein expression levels were analyzed by Western blot in EJ and T24 cells with LINC01605 overexpression and MMP9 knockdown. Data represent the mean ± S.D. from three independent experiments, *P<0.05, **P<0.01.

### Knockdown of LINC01605 impedes tumorigenesis *in vivo*

To further confirm the effect of LINC01605 expression on tumor growth *in vivo*, we subcutaneously implanted two groups of EJ cells with LINC01605 knockdown and control cells (sh-lnc01605 and NC, respectively) into the female nude mice. As indicated in Figure 6A,B, tumors from the sh-lnc01605 group grew dramatically slower than those from the NC group and the mean tumor weight of sh-lnc01605 group was also smaller than the NC group (Figure 6C). In addition, Ki-67 as a proliferation marker of tumors, was significantly decreased in the group of sh-lnc01605 (Figure 6D,E). Overall, these results presented that LINC01605 knockdown could markedly inhibit tumors growth *in vivo*.

**Figure 6:** Knockdown of LINC01605 impedes tumorigenesis *in vivo* (**A**) Representative pictures of tumor in EJ-NC and EJ-sh-lnc01605-2 cell-transplanted mice. (**B**,**C**) The tumor volume and weight were measured at the indicated weeks after mice were transplanted. (**D**) Cell proliferation was evaluated by Ki-67 immunohistochemistry in xenografs. (**E**) Statistical analysis of Ki-67 positive cells from panel. Data represent the mean ± S.D. from three independent experiments, *P<0.05, **P<0.01.

## Discussion

BC, characterized by its frequent recurrence and high mortality, remained to be a major clinical challenge, due to its poor long-term prognosis [26,27]. Accumulating data had suggested that lncRNAs, defined as non-coding RNA longer than 200 nts in length, could participate in the biology processes of cancers and meanwhile, various oncogenes and suppressor genes had been identified to be involved in the oncogenesis of BC [28–30]. Hence, it was imperative to find appropriate BC biomarkers which played an important role in the development and progression of disease. Based on the results of bioinformatics analysis, LINC01605, as one of the novel-found lncRNAs, was found to be highly expressed in BC tissues compared with matched normal tissues. Therefore, the present study focussed on the biological functions of LINC01605 and its potential clinical value in BC.

To the best of our knowledge, this was the first study to explore the relationship between LINC01605 and BC tumorigenesis and progression. LINC01605, a 2180-kb lncRNA, which maps to chromosome 8p11.23, was found to be highly expressed in four BC cell lines (EJ, T24, 253j, J82), compared with normal uroepithelial cells (SV-HUC-1). Besides, it was also frequently up-regulated in BC tissues and increased expression of LINC01605 in BC patients was correlated with higher histological grade, advanced TNM stage, and shorter overall survival in BC patients. Furthermore, EJ and T24 cell lines were chosen as cell models and the relative efficacy of silencing or overexpressing LINC01605 was confirmed by qRT-PCR. We could easily find that silencing LINC01605 could significantly reduce cell growth rate and colony formation efficiency, while overexpression of LINC01605 could markedly accelerate them. Similar outcomes could also be found in the migratory and invasive potential in BC cells. In addition, tumor xenografts mice model demonstrated that down-regulated LINC01605 could markedly inhibit tumor growth *in vivo*. Taken together, all these above data from different aspects suggested that LINC01605 might play an oncogenic role in BC.

With the advent of high-throughput sequencing methods as well as microarray analysis, it has facilitated identification of more novel lncRNAs, which have been demonstrated to play an important role in multiple tumors. Ye et al. [31] demonstrated that down-regulated linc00346 could inhibit the proliferation and migration of BC cell and induce cell cycle arrest and cell apoptosis. Wang et al. [32] indicated that LINC00312 could inhibit the migration and invasion of BC cells by targetting *miR-197-3p*. Zhao et al. [33] shed light on that by the mechanism of acting as a competing endogenous RNA, Linc00511 could regulate the expression of VEGFA through sponging hsa-*miR-29b-3p* in pancreatic ductal adenocarcinoma. In this study, we presented the oncogenic role of LINC01605 in BC by means of regulating its proliferation, migration, and invasion *in vitro* and *in vivo*.

Migration and invasion were two major events in the metastasis of cancer and there were many relevant signaling pathways involved in it [34]. Amongst them, the EMT, which referred to the conversion of epithelial cells into mesenchymal cells, played a crucial role in the progress of metastasis and it was characterized by its related proteins such as E-cadherin, N-cadherin, and vimentin [35,36]. The MMPs belonged to a family of zinc-dependent endopeptidases, which could degrade the extracellular matrix and had remarkable effects on tumor invasion and metastasis [36,37]. To further explore the underlying mechanism by which LINC01605 contributed to cell migration and invasion of BC, the relevant expression of EMT-related proteins and MMP9 was investigated. As exhibited in the results of Western blot, EMT-related proteins and MMP9 all had an obvious tendency. We could easily find that silencing could significantly down-regulate the expression of N-cadherin, Vimentin, β-catenin, and MMP9, while LINC01605 overexpression could markedly up-regulate their expression. Inspired by that, we supposed that LINC01605 might promote migration and invasion of BC by regulating EMT and extracellular matrix tissue degradation due to MMP9. Subsequently, down-regulating the protein level of MMP9 in the presence of LINC01605 could rescue the oncogenic role of the malignant behavior mediated by LINC01605 in BC, indicating that LINC01605 attributed its oncogenic role to the promotion of MMP9.

In summary, our study suggested that LINC01605 played its oncogene role by activating EMT signaling pathway and promoting the expression of MMP9. Future studies were required to explore its multiple mechanisms. Moreover, more and more non-coding RNAs and gene proteins had played a vital role in breast cancer, pancreatic cancer, and laryngeal carcinoma, alone and/or synergistically [38–40]. It would be interesting to investigate whether other non-coding RNAs or gene proteins also played a role, alone or coupled with LINC01605 in BC.

## Conclusion

In conclusion, our study suggested that LINC01605 was frequently highly expressed in BC cell lines and tissues and it could serve as a novel prognostic indicator for BC. *In vitro* and *in vivo* experiments further shed light on the promotion function of LINC01605 in BC proliferation and metastasis via activating the EMT signaling pathway and promoting the expression of MMP9. In other words, LINC01605 could become a novel therapeutic target and prognosis factor for the future treatment of BC.

## Abbreviations

BC: bladder cancer
EMT: epithelial–mesenchymal transition
lncRNA: long non-coding RNA
MMP: matrix metallopeptidase
qRT-PCR: quantitative real-time PCR
siMMP9: MMP9 small interference RNA
TCGA: The Cancer Genome Atlas
